The article "Oscillations of the baseline of solar magnetic field and solar irradiance on a millennial timescale" was retracted in 2020. Reasons: errors in the analysis; errors in the methods; errors in the results or conclusions.

# Oscillations of the baseline of solar magnetic field and solar irradiance on a millennial timescale

**DOI:** 10.1038/s41598-019-45584-3

**Published:** 2019-06-24

**Authors:** V. V. Zharkova, S. J. Shepherd, S. I. Zharkov, E. Popova

**Affiliations:** 1 Northumbria University, Department of Mathematics, Physics and Electrical Engineering, Newcastle upon Tyne, NE2 1XE UK; 2 University of Bradford, School of Engineering, Bradford, BD7 1DP UK; 3 University of Hull, Department of Physics and Mathematics, Kingston upon Hull, HU6 7RX UK; 4 Nasir al-Din al-Tusi Shamakhi Astrophysical Observatory Azerbaijan, AZ 1000 Pirqulu, Azerbaijan; 5 National Research University, Higher School of Economics, 101000 Moscow, Russia

**Keywords:** Solar physics, Solar physics

## Abstract

Recently discovered long-term oscillations of the solar background magnetic field associated with double dynamo waves generated in inner and outer layers of the Sun indicate that the solar activity is heading in the next three decades (2019–2055) to a Modern grand minimum similar to Maunder one. On the other hand, a reconstruction of solar total irradiance suggests that since the Maunder minimum there is an increase in the cycle-averaged total solar irradiance (TSI) by a value of about 1–1.5 *Wm*^−2^ closely correlated with an increase of the baseline (average) terrestrial temperature. In order to understand these two opposite trends, we calculated the double dynamo summary curve of magnetic field variations backward one hundred thousand years allowing us to confirm strong oscillations of solar activity in regular (11 year) and recently reported grand (350–400 year) solar cycles caused by actions of the double solar dynamo. In addition, oscillations of the baseline (zero-line) of magnetic field with a period of 1950 ± 95 years (a super-grand cycle) are discovered by applying a running averaging filter to suppress large-scale oscillations of 11 year cycles. Latest minimum of the baseline oscillations is found to coincide with the grand solar minimum (the Maunder minimum) occurred before the current super-grand cycle start. Since then the baseline magnitude became slowly increasing towards its maximum at 2600 to be followed by its decrease and minimum at ~3700. These oscillations of the baseline solar magnetic field are found associated with a long-term solar inertial motion about the barycenter of the solar system and closely linked to an increase of solar irradiance and terrestrial temperature in the past two centuries. This trend is anticipated to continue in the next six centuries that can lead to a further natural increase of the terrestrial temperature by more than 2.5 °C by 2600.

## Introduction

Understanding of solar activity is tested by the accuracy of its prediction. The latter became very difficult to derive from the observed sunspot numbers and to fit sufficiently close into the prediction of a few future solar cycles or even into a single solar cycle until the cycle is well progressed^1^. In many models there is a consistent disagreement for cycle 24 between the measured sunspot numbers and the predicted ones. This disagreement is a clear indication that there is something missing in the definition of solar activity by sunspot numbers, which are the collective product of many instruments and observers around the world. This discrepancy also indicates that the appearance of sunspots on the surface during a solar cycle is governed by the action of some physical processes of solar dynamo, which were not yet considered in the models. Moreover, it was first detected by Stix^2^ for cycle 22 and later confirmed by Zharkov *et al*.^3^ for cycle 23 that the polarity of solar background magnetic field is always opposite to the leading polarity of sunspots while timing and locations of sunspot appearance on the solar surface are, in fact, governed by this background magnetic field.

This research inspired us to investigate this solar background magnetic field s a new proxy of solar activity. In order to reduce dimensionality of any waves present in the observational data of the background magnetic field, Zharkova *et al*.^4^ explored a solar background magnetic field by applying Principal Component Analysis (PCA) to the low-resolution full disk magnetograms captured in cycles 21–23 by the Wilcox Solar Observatory. This approach revealed not one but two principal components (PCs) with the nearly-equal largest eigen values (strongest waves of solar magnetic oscillations) covering about 67% of the data by standard deviation^5,6^. The PCs are shown associated with two magnetic waves attributed to the poloidal magnetic field^6,7^ generated by a double dynamo with dipole magnetic sources in the inner and outer layers of the solar interior^8^. These waves are found to be asymmetric by default since they start in the opposite hemispheres while travelling with an increasing phase shift to the Northern hemisphere (in odd cycles) and to the Southern hemisphere (in even cycles)^4,6^. The maximum of solar activity for a given cycle (or double maximum for the double waves with a larger phase shift) occurs at the times when each of the waves approaches its maximum so that at the equal amplitudes the two waves can have resonant interaction. The hemisphere where it happens becomes the most active one, naturally accounting for the often-reported North-South asymmetry of solar activity in cycle 23^3,9^ and in a few other 11 year cycles^10–12^.

These two magnetic waves of poloidal field generated during a solar cycle by the electromotive force in the two layers (inner and outer) can be converted into two waves of the toroidal magnetic field associated with sunspots^7,13–15^. The summary curves of the two waves of poloidal magnetic field produce the two magnetic waves of toroidal magnetic field and their summary curve, whose modulus is closely associated with solar activity defined by the averaged sunspot numbers^5,6^. The existence of two waves in the poloidal (and toroidal) magnetic fields generated in two layers, instead of a single one used in the most prediction models, and the presence of a variable phase difference between the two waves can naturally explain the difficulties in predicting the solar activity (or our summary curve) with a single dynamo wave^16^.

The two magnetic waves generated by magnetic dipoles in two different layers of the solar interior generate with the electromotive force of solar dynamo^13^ toroidal magnetic fields, or magnetic loops which become sunspots on the surface. This interference is especially intense when the wave amplitudes become close, so that the waves can reach a resonance marking the maximum of solar activity for a given cycle. The hemisphere where these waves reach maxima, becomes the most active one. At the same time, the magnetic waves from the inner layer travel through the outer layer of solar interior to the solar surface and interfere with the magnetic waves generated in this outer layer. At some times the two waves, generated in inner and outer layers, appear to be in the anti-phase, causing a disruptive interference. This reduces dramatically the resulting wave magnitude and, thus, leads to significant reduction in production of toroidal fields, or sunspot numbers.

The resulting summary curve, which is linked to the solar activity curve defined by the averaged sunspot numbers^5^, restored backward for 3000 years shows about 9 grand cycles of 350–400 years, with the times of their grand minima having remarkable resemblance to those reported from the sunspot and terrestrial activity in the past millennia^17^: Maunder (grand) Minimum (1645–1715), Wolf grand minimum (1200), Oort grand minimum (1010–1050), Homer grand minimum (800–900 BC), combined with the warming periods: medieval (900–1200), Roman (400–10 BC) and other ones occurred between the grand minima. This approach allowed us to predict the modern grand solar minimum (GSM) approaching the Sun in 2020–2055^6^. This grand minimum offers a unique opportunity for the space scientists and all people of the planet to witness in many details the modern grand minimum and to understand better the nature of solar activity.

Although, it was noted^17,18^ that Sporer minimum (1460–1550) is not present in our summary curve, which instead during the same period of time shows a standard grand cycle, the previous one to the modern grand cycle (17–21 centuries). Zharkova *et al*.^17,18^ reasonably argued that Sporer minimum is an artifact of the strongly increased at that time background radiation on the Earth caused by the explosion of a very close (about 600–700 light years) supernova Vela Junior occurred in the southern sky. The radiation induced by this explosion for this period has not been considered in the background radiation required for the carbon dating method^19,20^ that could shift the dates by a few hundred years.

These two-wave magnetic field variations were tested with Parker’s two layer dynamo model with meridional circulation^6,7^ showing that the grand cycle variations of magnetic field are induced by a beating effect (with a period of 350–400 years) of the interference of magnetic waves generated in each layer. These variations are affected by the changes of solar dynamo numbers in each layer describing a joint action of solar differential rotation (Ω-effect) and radial shear (*α*-effect). It is assumed that the both dynamo waves are produced by dipole magnetic sources: one in the subsurface layer and the other deeply in the solar convection zone with the parameters in each layer to be rather different^6^. This difference led to two magnetic waves, similar to those derived with PCA (see Fig. 3 in Zharkova *et al*.^6^), which travel from one hemisphere to another^6^ with different but close frequencies and increasing phase shifts^7^ and producing the grand cycles of the similar durations and shapes as derived from the observations using PCA^4^.

The temporal and latitudinal patterns shown by two principal components defining dynamo waves generated in the inner and outer layers of the solar interior^6^ can naturally account for the difference in observed magnetic fluxes in the opposite hemispheres reported by Shetye *et al*.^12^. Since the two double dynamo waves travel with different phases, so that at a given moment they have different amplitudes (see Fig. 1 in Zharkova *et al*.^6^) that can explain a much larger magnetic flux observed in the Northern hemisphere than in the Southern one at the descending phase of cycle 23 and a reversed trend in the ascending phase of cycle 24 reported by Shetye *et al*.^12^. In addition, these two waves generated in different layers gain close but not equal frequencies^6^ because of different speeds of meridional circulation in each layer as suggested by Shetye *et al*.^12^, so that their interference naturally leads to a beating effect with the envelope oscillations (grand cycles) occurring at the frequency equal to a difference of frequencies of the individual waves^6^. The lengths of the individual grand cycles depend on a real time as shown in the summary curve of the solar activity extrapolated backward by two^6,21^ and three millennia^17,18^ making some grand cycles shorter with higher amplitudes and the other ones longer with smaller amplitudes.

**Figure 1:** Top plot: solar activity prediction backwards 3000 years with a summary curve (blue line) of the two principal components (PCs) of solar background magnetic field (SBMF)^6^ versus the reconstruction by Solanki *et al*.^27^ (red line). The summary curve is derived from the full disk synoptic maps of Wilcox Solar Observatory for cycles 21–23, the reconstructed solar activity curve^27^ was build by merging the sunspot activity curve (17–21 centuries) and a carbon-dating curve (before the 17 century). The bottom plot: the modulus summary curve of two PCs associated with averaged sunspot numbers^5^ calculated backward 120 (one hundred twenty) thousand years. The red line shows the baseline oscillations with a period of about 40 thousand years likely associated with the Earth’s axial tilt (obliquity) (see the text for further details).

All these derivations of the observed magnetic waves, or principal components, generated by dipole magnetic sources were carried out purely from the solar magnetic data assuming that the Sun is an isolated system generating its own waves by its own (dynamo) rules. However, Hays *et al*.^22^ shown that small planetary influences on the solar magnetism seen from the Earth can have long-term effects on the Earth’s climate. As established by Milankovich^22,23^ (see also https://en.wikipedia.org/wiki/Milankovitch_cycles) there are various aspects of the Earth movements in the solar system, which can affect the terrestrial climate changes over many thousand years^22,23^. For example, the Earth axis tilt is shown to affect the terrestrial temperature variations with season and their durations, while the Earth orbit eccentricity and different type of precession define long-term variations of the terrestrial temperature on a scale of 20, 40 and 100 thousand years as derived from the Antarctic glaciers^24–26^.

These orbital oscillations of the Earth rotation about the Sun strongly affect the solar irradiance and temperature on the Earth. Solar irradiance is accepted to be one of the important factors defining the temperature variations on the Earth and other planets as it is the main source of the energy. Reconstruction of the cycle-averaged solar total irradiance back to 1610 suggests that since the end of the Maunder minimum there was the increase of the irradiance by a value of about 1–1.5 *Wm*^−2^ ^27,28^, or about 3% of the total solar irradiance. This increase is correlated rather closely with the oscillations of the terrestrial temperature baseline^26^, which is found to steadily increasing since the Maunder minimum (e.g. recovering from the mini ice age). Although, it is not clear yet if this trend in the terrestrial temperature and solar irradiance is caused directly by the increased solar activity itself or by some other factors of the solar-terrestrial interaction in the whole solar system and human activities.

## Restoration of Double Dynamo Waves for the Past Hundred Millennia

As we shown earlier^5,6^, the resulting summary curve of the two magnetic waves detected with PCA can be used for prediction of a solar activity usually associated with the averaged sunspot numbers^5,6^. Let us explore this summary curve^6^, as approximation of the solar activity on larger timescale of hundred millennia.

In Fig. 1 we present 3000 years of the summary curve (top plot, blue curve) calculated backward from the current date, on which we overplotted the graph of the restored solar activity/irradiance derived by Solanki^27,28^ (top plot, red curve). The solar irradiance curve prior 17 century was restored from the carbon isotope Δ^14^C abundances in the terrestrial biomass merged in 17 century till present days with the solar activity curve derived from the observed sunspot numbers.

It can be noted that in many occasions the summary curve plotted backward for 3000 years in Fig. 1 reveals a remarkable resemblance to the sunspot and terrestrial activity reported for these 3000 years from the carbon isotope dating^27^. The summary curve shows accurately the recent grand minimum (Maunder Minimum) (1645–1715), the other grand minima: Wolf minimum (1300–1350), Oort minimum (1000–1050), Homer minimum (800–900 BC); also the Medieval Warm Period (900–1200), the Roman Warm Period (400–150 BC) and so on. These grand minima and grand maxima reveal the presence of a grand cycle of solar activity with a duration of about 350–400 years that is similar to the short term cycles detected in the Antarctic ice^25,26^. The 11/22 and 370–400 year cycles were also confirmed in other planets by the spectral analysis of solar and planetary oscillations^29,30^. The next Modern grand minimum of solar activity is upon us in 2020–2055^6^.

Zharkova *et al*.^6^ pointed out that longer grand cycles have a larger number of regular 11 year cycles inside the envelope of a grand cycle but their amplitudes are lower than in shorter grand cycles. This means that there are significant modulations of the magnetic wave frequencies generated for different grand cycles in these two layers: a deeper layer close to the bottom of the Solar Convective Zone (SCZ) and shallow layer close to the solar surface whose physical conditions derive the dynamo wave frequencies and amplitudes. The larger the difference between these frequencies the smaller the number of regular 22 years cycles inside the grand cycle and the higher their amplitudes. Later Popova *et al*.^21^ have also shown that the reduced solar activity during Dalton minimum (1790–1820), which was weakly present in the summary curve for dipole sources^6^, is reproduced much closer to the observations of averaged sunspot activity by consideration of the quadruple components of magnetic waves, the next two eigen vectors obtained with PCA^4^, produced by quadruple magnetic sources.

In addition, in Fig. 1 (bottom plot) we present the summary curve simulated for 100 000 years backwards from now (blue line), on which we over-plotted the averaged baseline curve (red curve) filtering large cycle oscillations with a running averaging filter of 25 thousand years. This plot reveals the baseline oscillations of about 40,000 (forty thousand) years (see the periodic function appearing between 20 K and 60 K years in the bottom plot). They are likely to be the oscillations caused by the Earth axis tilt (obliquity)^22,23^ e.g. by precession of the tilt of the axis of Earth’s rotation relative to the fixed stars^23^, or the variations of the Earth axis tilt between 22.1° and 24.5° (the current tilt is 23.44°). This Earth obliquity effect is incorporated into the summary curve derived by us from the solar magnetic observations. This indicates that the measurements of a magnetic field of the Sun from the Earth, or from the satellites on the orbit close to Earth, contain also the orbital effects of the Earth rotation about the Sun and of any other motion by the Sun itself, which we intend to explore further in the sections below.

### Detection of the baseline oscillations of solar magnetic field

In Fig. 2 we present 20 000 years of the summary curve (between 70 and 90 thousand years backward), in which, in addition to the grand cycles of 350–400 years of solar activity, there are also indications of larger super-grand cycles marked by the vertical lines (the top plot). By comparing in Fig. 2 (top plot) the semi-similar features (between the vertical lines) of the repeated five grand cycles of total with a duration of about 2000–2100 years, one can see a striking similarity of the shapes of these 5 grand cycles, which are repeated about 9 (nine) times during the 20 000 years.

**Figure 2:** Top plot: the summary curve of two magnetic field waves, or PCs, calculated backward ten thousand years from the current time. The vertical lines define the similar patterns in five grand cycles repeated every 2000–2100 years (a super-grand cycle). Bottom plot: the oscillations of the summary curve (cyan line) calculated backward from 70 K to 90 K years overplotted by the oscillations of a magnetic field baseline, or its zero line (dark blue line) with a period of about 1950 ± 95 years. The baseline oscillations are obtained with averaging running filter of 1000 years from the summary curve suppressing large scale cycle oscillations. The left Y-axis shows the scale of variations of the baseline magnetic field, while the right Y-axis presents the scale of variations of the summary curve.

In order to understand the nature of these super-grand oscillations and to derive the exact frequency/period of this super-grand cycle, let us filter out large oscillations of 11/22 year solar cycles with the running averaging filter (1000 years). The resulting baseline oscillations are shown by a dark blue curve in Fig. 2 (bottom plot) over-plotted on the summary curve (light blue curve) taken from the summary curve calculated backwards between 90 and 70 thousand years. For a comparison, the left Y-axis gives the range of variations of the baseline curve (−10, 10) while the right side Y-axis produces the same for the summary curve (−500, 500). The baseline variations are, in fact, the variations of the zero-line of the summary curve, which are too small to observe on this curve without filtering large-scale oscillations of 11 year cycles.

It is evident that the dark blue line in Fig. 2 (bottom plot) shows much (50 times) smaller oscillations of the baseline of magnetic field with a period of years, which is incorporated into the magnetic field measurements of the summary curve (light blue curve). The baseline oscillations show a very stable period of 2000–2100 years occurring during the whole duration of simulations of 120 thousand years, for which the summary curve was calculated. This means that this oscillation of the baseline magnetic field has to be induced by a rather stable process either inside or outside the Sun. This baseline oscillation period is very close to the 2100–2400 year period reported from the other observations of the Sun and planets^29–31^.

To understand the nature of these oscillations, we decided to compare these oscillations with the solar irradiance curve derived for the past 10000 years by Solanki, Krivova *et al*.^27,28^ as presented for 3000 years in Fig. 1 (top plot, red curve). In Fig. 3 the irradiance curve by Krivova and Solanki^27,28^ was plotted for the current and the past grand cycles as follows: the summary curve of magnetic field (light blue line), the oscillations of the baseline (dark blue line) and the restored solar irradiance^27,28^ (magenta line), which was was slightly reduced in magnitude in the years 0–1400, in order not to obscure the baseline oscillations. The dark rectangle indicates the position of Maunder Minimum (MM) coinciding with the minimum of the current baseline curve and the minimum of solar irradiance. After the MM the baseline curve is shown growing for the next 1000 years (e.g. until 2600). During the current years the solar irradiance curve^27,28^ follows this growth of the baseline (with a correlation coefficient about 0.68).

**Figure 3:** Top plot: the close-up view of the oscillations of the baseline magnetic field (dark blue curve) in the current and past millennia with a minimum occurring during Maunder Minimum (MM). The irradiance curve (magenta line) presented from Krivova and Solanki^27,28^ overplotted on the summary curve of magnetic field (light blue curve)^6^. Note the irradiance curve is slightly reduced in magnitude in the years 0–1400 to avoid messy curves. The dark rectangle indicates the position of MM coinciding with the minimum of the current baseline curve and the minimum of the solar irradiance^27,28^. The scale of the baseline variations are shown on the left hand side of Y axis, the scale of the summary curve - on the right hand side. Bottom plot: variations of the Earth temperature for the past 140 years derived by Akasofu^26^ with the solid dark line showing the baseline increase of the temperature, blue and red areas show natural oscillations of this temperature caused by combined terrestrial causes and solar activity. The increase of terrestrial temperature is defined by 0.5 °C per 100 years^26^.

For the further information we present in Fig. 3 (bottom plot) the variations of the Earth temperature for the past 140 years as derived by Akasofu^26^ with the solid dark line showing the baseline increase of the temperature, blue and red areas show natural oscillations of this temperature caused by combined terrestrial causes and solar activity. The trend derived by Akasofu^26^ shows the increase of the terrestrial temperature by 0.5 °C per 100 years. This temperature growth is also expected to continue in the next 600 years until 2600. Although, if it follows the baseline curve, this growth could not be linear as it was at the early years shown in the Akasofu’s curve^26^ but will have some saturation closer to the maximum as any periodic functions (sine or cosine) normally have.

### Links of the baseline oscillations with solar inertial motion (SIM)

Principal components and their summary curve were detected from the solar background magnetic field oscillations produced in the Sun. Large part of these oscillations related to 11 year solar cycle and 350–400 year grand cycle are well accounted for by the solar dynamo waves generated dipole magnetic sources in inner and outer layers^6^. They can explain the magnetic field oscillations with a grand cycle by the beating effects of the two waves generated these two layers. However, it is rather difficult to find any mechanism in the solar interior that can explain much weaker and longer oscillations of the baseline of magnetic field. Therefore, we need to look for some external reasons for these oscillations.

Kuklin^32^ first suggested that solar activity on a longer timescale can be affected by the motion of large planets of the solar system. This suggestion was later developed by Fairbridge^31^, Charvatova^33^ and Palus^34^ who found that the Sun, as a central star of the solar system, is a subject to the inertial motion around the barycenter of the solar system induced by the motions of the other planets (mostly large planets, e.g. Neptune, Jupiter and Saturn).

Solar inertial motion (SIM) is the motion of the Sun around this barycenter of the solar system as shown in Fig. 4 reproduced from the paper by Richard Mackey^35^. Shown here are three complete orbits of the Sun, each of which takes about 179 years. Each solar orbit consists of about eight, 22-year solar cycles^35^. The total time span shown in Fig. 4 is, therefore, three 179-year solar cycles^31^, for about 550–600 years. The Sun rotates around the solar system barycenter inside the circle with a diameter of about Δ = 4.3*R*_*Sun*_, or Δ = 29 910 km, where *R*_*Sun*_ is a solar radius. This schematic drawing illustrates sudden shifts in the solar inertial motion (SIM) as the Sun travels in an epitrochiod-shaped orbit about the center-of mass of the solar system.

**Figure 4:** Left plot: the example of SIM trajectories of the Sun about the barycenter calculated from 1950 until 2100^34^. Right plot: the cone of expanding SIM orbits of the Sun^35^ with the top showing 2D orbit projections similar to the left plot. Here there are three complete SIM orbits of the Sun, each of which takes about 179 years. Each solar orbit consists of about eight, 22-year solar cycles^35^. The total time span is, therefore, three 179-year solar cycles^31^, or about 600 years. Source: Adapted from Mackey^35^. Reproduced with permission from the Coastal Education and Research Foundation, Inc.

The SIM has very complex orbits induced the trifall positions of large planets achieved for different planet configurations changing approximately within 370 years as indicated by Charvatova^33^. She also claimed that there is a a larger period of 2100–2400 years related to the full cycle of the planet positions in their rotation around the Sun^36^ (see Fig. 5 from Charvatova’s paper). Since the SIM occurs for the Sun observed from the Earth, we believe, only the SIM can define the weak oscillations of the baseline of solar magnetic field reported above.

**Figure 5:** Schematic presentation of the solar inertial motion (SIM) about the barycenter of the solar system defined by the gravitational forces of large planets in the plane of ecliptics (the top plane in Fig. 4) for different time intervals shown in the top of each sub-figure (reproduced from Charvatova^36^. The location of the Sun at the end of the period is shown by the yellow circles. Top row represent the ordered SIM affected by symmetric positions of large planets with respect to the Sun, while the bottom row shows the disorganized SIM with more random positions of large planets.

Although, unlike Fairbridge^31^ and Charvatova^33^, we do not propose a replacement of the solar dynamo role in solar activity with the effects of large planets, or solar inertial motion. This replacement would be very unrealistic from the energy consideration^37^ because the tidal effects of the planets are unable to cause a direct effect on the dynamo wave generation in the bottom of solar convective zone (SCZ).

However, in the light of newly discovered double dynamo effects in the solar interior^6^ the planets can surely perturb properties of the solar interior governing the solar dynamo in the outer layer, such as solar differential rotation, or Ω-effect, governing migration of a magnetic flux through the outer layer to its surface, and those of *α* effect, that can change the velocity of meridional circulation. This leads to the dynamo waves in this outer layer with the frequency slightly different from that than in the inner layer, and, thus to the beating effects caused by interference of these two waves and to grand cycles discussed above^6^.

Although, Abreu *et al*.^38^ suggested that the tidal forces of large planets can excite gravity waves at the tachocline, which can propagate to the surface balanced by buoyancy of the solar interior^39,40^ and insert a net tidal torque in the small region between the tachocline and radiative zone. At the same time the shape of tachocline was inferred from helioseismic observations with prolate geometry to show the ellipticity 1000 times higher than at the photospheric level^41^.

Using this finding, Abreu *et al*.^38^ suggested that a possible planetary torque can appear from the nonspherical tachocline and modulate the dynamo waves properties generated there (Abreu *et al*., 2012). The authors used either ^10^*Be* or ^14^*C* isotope production rates of the terrestrial proxies to derive the various periods of solar and terrestrial activity using wavelet analysis and found the periods close to 370 and 2100 years reported above. Although, the periods of this activity found by Abreu *et al*.^38^ were later objected by Cameron and Shussler^42^, who argued that these activity periods are random and do not have a real causal force. This dialog demonstrated that the absence of long-term solar data was the obstruction for the accurate detection of shorter periods of the solar-terrestrial activity.

However, a detection with PCA of the solar background magnetic field^4,6^ and the HMI helioseismic observations^8^ of two layers in the solar interior with different directions and speeds of meridional circulation where two dynamo waves can be generated either by dipole^6^ or dipole plus quadruple^21^ magnetic sources lifts these rather rigid requirements for the planetary torque to act very deeply inside the Sun at its tachocline. Instead, the planetary torque can affect differently the buoyancy and differential rotation of the convective zone in the outer layers in both hemispheres, thus, producing there rather different *α*- and Ω-effects and different velocities of meridional circulation compared to those in the inner layer near the bottom of the tachocline.

These parameters, in turn, are likely to be the effective contributors governing the frequencies and phases of the dynamo waves in the outer layer, thus, producing the resulting beating frequencies obtained from the summary wave caused by these two wave interference.

### Effects of SIM on a temperature in the terrestrial hemispheres

It was indicated by Shirley *et al*.^43^ that the solar irradiance caused by SIM can be increased by up 3.5% in the closest point to the Earth and decreased by the same amount in the most distant point. And these closest and most distant points vary in time from the aphelion (summer solstice) to perihelion (winter solstice) with a period of about 2100–2400 years^36^.

In order to understand how this SIM motion would affect the solar irradiance at the Earth orbit, let us look at the drawing of the Earth motion around the Sun (Fig. 6)^44,45^. If the Sun was stationary and located in the focus of the Earth orbit, then the solar irradiance and, thus, the seasons on the Earth are defined by the position of our planet on the orbit around the Sun. In the aphelion (1.53 × 10^8^ km from the focus where the Sun is located, 21–24 June, position 1, there is a summer in the Northern hemisphere and winter in the Southern hemisphere. While in the perihelion (1.47 × 10^8^ km from the Earth orbit focus, 21–24 December, position 2, there is a summer in the Southern and winter in the Northern hemispheres. The seasons are caused by the increase or reduction of the solar irradiance caused, in turn, by the inclination of the Earth’s axis towards or from the Sun.

**Figure 6:** The schematic Earth orbit about the Sun^48^ (shown not to the real scale of the Sun and Earth) with the indication of the solar irradiance at different phases of the orbit^44,45^. The arrows coming from the centre of the Sun in two perpendicular directions are symbolic axis of the Earth orbital motion: vertical one is shorter and the horizontal one is slightly longer according to the Earth orbit eccentricity. The other arch arrows are also symbolic showing the direction of the Earth rotation about the Sun (anti-clockwise). The Earth axis is shown by the thin lines coming from the North and South poles, the dark parts of the Earth disk show the night, and the blue ones show the day. The Earth latitudes are shown by the light lines on the disk, while the current angle of the Earth axis inclination from the perpendicular to the ecliptics is shown in the winter solstice (the right disk).

Since the Sun moves around the solar system barycenter, it implies that it also shifts around the main focus of the Earth orbit being either closer to its perihelion or to its aphelion. If the Earth rotates around the Sun undisturbed by inertial motion, then the distances to its perihelion will be 1.47 × 10^8^ km and to it aphelion 1.52 × 10^8^ km. The solar inertial motion means for the Earth that the distance between the Sun and the Earth has to significantly change (up to 0.02 of a.u) at the extreme positions of SIM, and so does the average solar irradiance, which is inversely proportional to the squared distance between the Sun and Earth.

If during SIM the Sun moves closer to perihelion and the spring equinox (positions 2), thus increasing the Earth orbit eccentricity, the distance between the Sun and Earth will be the shortest at perihelion approaching about 1.44 × 10^8^ km while at aphelion it will increase to 1.55 × 10^8^ km. This means at these times the Earth would receive higher than usual solar irradiance (that can lead to higher terrestrial temperatures)^26,43,44^, while approaching its perihelion during its winter and spring (warmer winters and springs in the Northern hemisphere and summers and autumns in the Southern one). At the same time, when the Earth moves to its aphelion, the distance between the Earth and Sun is increased because of the SIM resulting in the reduced solar irradiance during summer and autumn in Northern and winter/spring in the Southern hemispheres. This scenario with the solar irradiance and terrestrial temperature was likely to happen during the millennium prior the Maunder Minimum.

If the Sun moves in its SIM closer to Earth’s aphelion (position 1) decreasing the Earth orbit eccentricity and to the autumn equinox as it is happening in the current millennium starting from Maunder Minimum, then the distance between Sun and Earth at the aphelion will become shorter approaching 1.49 × 10^8^ km during the summer in the Northern and winter in the Southern hemispheres, and longer at the perihelion approaching 1.50 × 10^8^, or during a winter in the Northern and summer in the Southern hemispheres. Hence, at this SIM position of the Sun, the Earth in aphelion should receive higher solar irradiance (and temperature)^43,44^ during the Northern hemisphere summers and Southern hemisphere winters. When the Earth moves to its perihelion, the distance to the Sun will become longer and thus, the solar irradiance will become lower leading to colder winters in the Northern hemisphere and colder summers in the Southern one. This is what happening in the terrestrial temperature in the current millennium starting since Maunder minimum and lasting until ≈2600.

Hence, it is evident that the oscillations of the solar inertial motion around the barycentre of the solar system should produce the very different variations of solar irradiance in each hemisphere of the Earth at different seasons. These variations occur in addition to any other variations of the solar irradiance caused by larger variations of the solar activity itself caused by the action of solar dynamo. Furthermore, Dikpati *et al*.^46^ shown that under certain conditions the magnetic field can be conserved by the dynamo machine below the solar convective zone^46^ that can potentially contribute to the increase of the baseline magnetic field by bringing this conserved field upwards by the SIM. Currently, the solar system is at the SIM phase when the Sun moves towards the aphelion (position 1). This is expected to lead to a steady increase for another 600 years of the baseline magnetic field and, thus, the summer temperature in the Northern hemisphere and winter temperature in the Southern one and decrease of the winter temperature in the Northern and summer temperature in the Southern hemispheres.

The increase of the solar irradiance at these times is expected to lead to the increase of the terrestrial temperature^43,44^ in the Northern hemisphere where the most solar observatories measuring the terrestrial temperature are located. Since Akasofu^26^ derived the rate of the temperature increase in the past centuries to be about 0.5C per 100 years (see Fig. 3, bottom plot). Therefore, with a very conservative extrapolation of this temperature into the next six centuries, following the parabola of the baseline wave caused by SIM, we expect an increase of the terrestrial temperature in the Northern hemisphere from the current magnitude by about 2.5C or slightly higher. This increase is caused solely by the Sun’s rotation about the barycenter of the solar system as it is shown in Fig. 3, top plot. Given the fact that these temperature variations have already happened on the Earth many thousand times in the past, one expects the Earth-Sun system to handle this increase in its usual ways. Of course, any human-induced contributions can make this increase more unpredictable and difficult to handle if they will override the effects on the temperature induced by the Sun.

We have to emphasize that there still will be, of course, the usual magnetic field and temperature oscillations caused by standard solar activity cycles of 11 and 350–400 years as reported before^6^ occurring on top of these baseline oscillations caused by SIM. As result, the solar irradiance and terrestrial temperature are expected to oscillate around this baseline for the next 600 years while increasing during the maxima of 11 year and 350 year solar cycles and decreasing during their minima, similarly to the natural temperature variations oscillating about the temperature baseline shown by black line in the plot by Akasofu^26^ (see Fig. 3, bottom plot and Akasofu’s Fig. 9^26^). However, during the next two grand solar minima, which are expected to occur in 2020–2055 (Modern grand solar minimum lasting for 3 solar cycles) and in 2370–2415 (future grand solar minimum lasting for 4 cycles) (see Fig. 3 in Zharkova *et al*.^6^) a decrease of the terrestrial temperature is expected to be similar to those during the Maunder Minimum and, definitely, substantially larger than natural temperature fluctuations shown in the Akasofu’s plot^26,47^. Note, these oscillations of the estimated terrestrial temperature do not include any human-induced factors, but only the effects of solar activity itself and solar inertial motion.

## Conclusions

Until recently, solar activity was accepted to be one of the important factors defining the temperature on Earth and other planets. In this paper we reproduced the summary curve of the solar magnetic field associated with solar activity^5,6^ for the one hundred thousand years backward by using the formulas describing the sum of the two principal components found from the full disk solar magnetograms. In the past 3000 years the summary curve shows the solar activity for every 11 years and occurrence of 9 grand solar cycles of 350–400 years, which are caused by the beating effects of two magnetic waves generated by solar dynamo at the inner and outer layers inside the solar interior with close but not equal frequencies^6^.

The resulting summary curve reveals a remarkable resemblance to the sunspot and terrestrial activity reported in the past millennia including the significant grand solar minima: Maunder Minimum (1645–1715), Wolf minimum (1200), Oort minimum (1010–1050), Homer minimum (800–900 BC) combined with the grand solar maxima: the medieval warm period (900–1200), the Roman warm period (400–10BC) etc. It also predicts the upcoming grand solar minimum, similar to Maunder Minimum, which starts in 2020 and will last until 2055.

A reconstruction of solar total irradiance suggests that there is an increase in the cycle-averaged total solar irradiance (TSI) since the Maunder minimum by a value of about 1–1.5 *Wm*^−2^ ^27^. This increase is closely correlated with the similar increase of the average terrestrial temperature^26,43^. Moreover, from the summary curve for the past 100 thousand years we found the similar oscillations of the baseline of magnetic field with a period of 1950 ± 95 years (a super-grand solar cycle) by filtering out the large-scale oscillations in 11 year cycles. The last minimum of a super-grand cycle occurred at the beginning of Maunder minimum. Currently, the baseline magnetic field (and solar irradiance) are increasing to reach its maximum at 2600, after which the baseline magnetic field become decreasing for another 1000 years.

The oscillations of the baseline of solar magnetic field are likely to be caused by the solar inertial motion about the barycentre of the solar system caused by large planets. This, in turn, is closely linked to an increase of solar irradiance caused by the positions of the Sun either closer to aphelion and autumn equinox or perihelion and spring equinox. Therefore, the oscillations of the baseline define the global trend of solar magnetic field and solar irradiance over a period of about 2100 years. In the current millennium since Maunder minimum we have the increase of the baseline magnetic field and solar irradiance for another 580 years. This increase leads to the terrestrial temperature increase as noted by Akasofu^26^ during the past two hundred years. Based on the growth rate of 0.5 C per 100 years^26^ for the terrestrial temperature since Maunder minimum, one can anticipate that the increase of the solar baseline magnetic field expected to occure up to 2600 because of SIM will lead, in turn, to the increase of the terrestrial baseline temperature since MM by 1.3 °C (in 2100) and, at least, by 2.5–3.0 °C (in 2600).

Naturally, on top of this increase of the baseline terrestrial temperature, there are imposed much larger temperature oscillations caused by standard solar activity cycles of 11 and 350–400 years and terrestrial causes. The terrestrial temperature is expected to grow during maxima of 11 year solar cycles and to decrease during their minima. Furthermore, the substantial temperature decreases are expected during the two grand minima^47^ to occur in 2020–2055 and 2370–2415^6^, whose magnitudes cannot be yet predicted and need further investigation. These oscillations of the estimated terrestrial temperature do not include any human-induced factors, which were outside the scope of the current paper.
